RETRACTED

# Correlations of Ezrin Expression with Pathological Characteristics and Prognosis of Osteosarcoma: A Meta-Analysis

**DOI:** 10.1155/2014/837543

**Published:** 2014-11-27

**Authors:** Da-Hang Zhao, Jiang Zhu, Wen-Bo Wang, Feng Dong, Qiao Zhang, Hong-Wu Fan, Jing-Zhe Zhang, Yong-Ming Wang

**Affiliations:** ^1^3rd Department of Orthopedics, The First Affiliated Hospital of Harbin Medical University, No. 23 Youzheng Street, Harbin 150001, China; ^2^4th Department of Orthopedics, The Fourth Affiliated Hospital of Harbin Medical University, Harbin 150001, China; ^3^Department of Orthopedics, China Japan Union Hospital of Jilin University, Changchun 130033, China

## Abstract

We conducted a meta-analysis to comprehensively evaluate the correlations of ezrin expression with pathological characteristics and the prognosis of osteosarcoma. The MEDLINE (1966–2013), the Cochrane Library Database, EMBASE, CINAHL, Web of Science (1945–2013), and the Chinese Biomedical Database were searched without language restrictions. Meta-analyses conducted using STATA software were calculated. Ten studies met the inclusion criteria, including 459 patients with osteosarcoma. Meta-analysis results illustrated that ezrin expression may be closely associated with the recurrence of osteosarcoma or metastasis in osteosarcoma. Our findings also demonstrated that patients with grade III-IV osteosarcoma showed a higher frequency of ezrin expression than those with histological grade I-II osteosarcoma. Furthermore, we found that patients with positive expression of ezrin exhibited a shorter overall survival than those with negative ezrin expression. The results also indicated that positive ezrin expression was strongly correlated with poorer metastasis-free survival. Nevertheless, no significant relationships were observed between ezrin expression and clinical variables (age and gender). In the current meta-analysis, our results illustrated significant relationships of ezrin expression with pathological characteristics and prognosis of osteosarcoma. Thus, ezrin expression could be a promising marker in predicting the clinical outcome of patients with osteosarcoma.

## 1. Introduction

Osteosarcoma, a type of malignant tumor originating from primitive bone-forming mesenchymal cells, is the most prominent primary bone tumor that mainly develops in children and adolescents [1, 2]. Osteosarcoma is the eighth most common type of childhood cancer, comprising 2.4% of all malignant tumors in children and young adult patients, and the mortality of osteosarcoma has been declining by about 1.3% per year [3]. Furthermore, the incidence rates of osteosarcoma increase rapidly in two periods: the first peak during adolescence (10~14-year-old) and the second peak in older adulthood (over 65 years old) [3]. As a complicated disease, osteosarcoma results from interactions between genetic and environmental factors [2, 4]. A number of epidemiological studies have demonstrated that a variety of environmental factors may contribute to the development of osteosarcoma, including age, gender, ethnicity, growth and height, and finally physical, chemical, and biological agents [4, 5]. In addition to those environmental factors, some studies showed that genetic factors may also play a more important role in the pathogenesis of osteosarcoma in recent years [6, 7]. Nowadays, many studies have suggested that ezrin may be implicated in the development and prognosis of osteosarcoma [8, 9].

RETRACTED

Ezrin, also identical to cytovillin or villin 2, is a component of cell-surface structures belonging to the ezrin/radixin/moesin (ERM) protein family that acts as a membrane organizer and linker between the plasma membrane and cytoskeleton [10, 11]. Ezrin is suggested to be involved in cell adhesion to the extracellular matrix and in cell-cell interactions, receptor tyrosine-kinase signaling, signal transduction through Rho GTPase, and interactions with the Akt-mediated cellular apoptotic machinery [12, 13]. Recently, there is evidence supporting that ezrin expression was connected with pathological characteristics and the clinical outcome of osteosarcoma [13, 14]. In general, ezrin connection allows the cell to interact with its microenvironment, facilitating intracellular signal transduction, which is responsible for the role of ezrin in tumor metastasis [14]. However, the alteration of ezrin expression mediates many changes in the metastasis-associated cell-surface signals and thereby may contribute to the invasion and metastasis of osteosarcoma [15]. On the other hand, ezrin protein currently has been identified as a potential and independent negative prognostic marker for event-free and overall survival in high-grade osteosarcoma [8, 12]. A reasonable explanation may be that ezrin is capable of interacting with integrins, which promotes the interaction of tumor cells that stimulate tumor adhesion and invasiveness [16]. Specifically, such ligand binding to integrins may lead to association with focal adhesion kinase (FAK) and recruitment of actin filaments regulated by the small GTPase RhoB, which play a crucial role in tumor resistance to chemotherapy [13]. Therefore, we hypothesized that the expression of ezrin is promising as a biomarker to predict the invasion, metastasis, and prognosis of osteosarcoma [17, 18]. In recent decades, abundant studies have revealed that expression of ezrin may be significantly related to the pathological characteristics and prognosis of osteosarcoma [15, 19], while there also existed inconsistent results reported in other studies [20, 21]. In this regard, we carried out this meta-analysis to evaluate the correlations of ezrin expression with the pathological characteristics and prognosis of osteosarcoma.

RETRACTED

## 2. Materials and Method

### 2.1. Literature Search and Selection Criteria

The MEDLINE (1966–2013), the Cochrane Library Database (Issue 12, 2013), EMBASE (1980–2013), CINAHL (1982–2013), Web of Science (1945–2013), and the Chinese Biomedical Database (CBM) (1982–2013) were searched without language restrictions. We used the following keywords and MeSH terms in conjunction with a highly sensitive search strategy: [“ezrin” or “phosphoprotein p81” or “villin-2” or “cytovillin” or “villin 2 protein”] and [“osteosarcoma” or “osteocarcinoma” or “bone neoplasms” or “cancer of the bone”]. We also conducted a manual search to find other potential articles based on references identified in the individual articles.

The following criteria were for the eligibility of included studies: (1) the study design must be a clinical cohort study that focused on the relationships of ezrin expression with pathological characteristics and prognosis of osteosarcoma; (2) all patients met the diagnostic criteria for osteosarcoma; (3) the study must provide sufficient information about expression levels of ezrin. The articles that did not meet our inclusion criteria must be excluded. The most recent or the largest sample size publication was included when the authors published several studies using the same subjects.

### 2.2. Data Extraction and Methodological Assessment

Data was systematically extracted by two authors from each included study by using a standardized form. The form used for data extraction documented the most relevant items including language of publication, publication year of article, the first author's surname, geographical location, design of study, sample size, the source of the subjects, protein expression levels, source of samples, detection of protein, and so forth.

Methodological quality was evaluated separately by two observers using the Newcastle-Ottawa Scale (NOS) criteria [27]. The NOS criteria included three aspects: (1) subject selection: 0–4; (2) comparability of subject: 0–2; (3) clinical outcome: 0–3. NOS scores ranged from 0 to 9; and a score ≥7 indicates a good quality.

### 2.3. Statistical Analysis

Meta-analysis was performed with the use of the STATA statistical software (Version 12.0, Stata Corporation, College Station, TX, USA). Odds ratios (OR), a hazard ratio (HR), and a 95% confidence interval (95% CI) were calculated as estimates of the impact of ezrin expression on pathological characteristics and prognosis of osteosarcoma. The *Z*-test was used to estimate the statistical significance of pooled ORs and HRs. Heterogeneity among studies was estimated by Cochran's *Q*-statistic and *I* ^2^ tests [28]. If *Q*-test shows a *P* < 0.05 or *I* ^2^ test exhibits >50%, which indicates significant heterogeneity, the random-effect model was conducted, or else the fixed-effects model was used. We also explored reasons for heterogeneity using metaregression and subgroup analyses. In order to evaluate the influence of single studies on the overall estimate, a sensitivity analysis was performed. Funnel plots and Egger's linear regression test were applied to investigate publication bias [29].

RETRACTED

## 3. Results

### 3.1. Study Selection and Characteristics of Included Studies

Initially, the highly sensitive search strategy identified 102 articles. We reviewed the titles and abstracts of all articles and excluded 40 articles; then we systematically reviewed full texts and 47 articles were further excluded (Figure 1). Finally, 10 clinical cohort studies with a total of 459 patients with osteosarcoma met our inclusion criteria for qualitative data analysis [14, 15, 19–26]. Publication years of the eligible studies ranged from 2006 to 2013. Distribution of the number of topic-related literatures in the electronic database during the last decade is shown in Figure 2. Overall, 7 studies were conducted among Asian and 3 among Caucasians. Five genotyping methods were utilized in the current meta-analysis, including labeled streptavidin-biotin method (LSAB), EnVision, MaxVision, avidin-biotin complex (ABC), and streptavidin-perosidase (SP) methods. We summarized the study characteristics and methodological quality in Table 1.

### 3.2. Quantitative Data Synthesis

Our results revealed that ezrin expression might be closely associated with recurrence of osteosarcoma or metastasis in osteosarcoma (Recurrence/Metastasis: OR = 12.96, 95% CI = 5.20~32.31, *P* < 0.001) (Figure 3). Our findings also demonstrated that patients with grade III-IV osteosarcoma showed a higher frequency of ezrin expression than those with grade I-II osteosarcoma (OR = 2.49, 95% CI = 1.33~4.69, *P* = 0.005). Furthermore, we found that patients with positive expression of ezrin exhibited a shorter overall survival than those with negative ezrin expression (OR = 2.30, 95% CI = 0.03~4.57, *P* = 0.047). The results also indicated that positive ezrin expression was strongly correlated with poorer metastasis-free survival (OR = 2.54, 95% CI = 1.04~4.03, *P* = 0.001) (Figure 3). Nevertheless, no significant relationships were observed between ezrin expression and clinical variables (age and gender) (all *P* > 0.05).

RETRACTED

Sensitivity analysis was performed to assess the influence of each individual study on the pooled estimates by omitting individual studies. The outcomes indicated that the overall pooled ORs and HRs could not be affected by a single study (Figure 4). Funnel plots demonstrated no evidence of obvious asymmetry existing (Figure 5). Egger's test also did not display strong statistical evidence for publication bias (all *P* > 0.05).

## 4. Discussion

In the current meta-analysis, we aimed to investigate whether ezrin expression may affect the pathological characteristics and prognosis in patients with osteosarcoma. The results of our meta-analysis showed significant correlations of ezrin expression with recurrence of osteosarcoma and metastasis in osteosarcoma, implying that expression of ezrin protein may be a novel mediator in promoting tumor cell invasion and metastasis in osteosarcoma. Nevertheless, the precise mechanisms by which the enhanced expression of ezrin protein leads to an aggressive invasion and metastasis in the progression of osteosarcoma are still largely unknown. It is well established that ezrin is both a key plasma membrane-cytoskeleton crosslinker and the binding partner of a plethora of molecules, and it is also responsible for the adhesion, migration, and invasion to cells or substrates during the multistep regulatory system [30]. Furthermore, ezrin also plays a critical role in signal transduction through the activation of small GTPase Ras [31]. In this regard, alternation in ezrin expression may in turn influence metastasis in osteosarcoma [32]. We therefore hypothesized that the increased expression of ezrin protein, by providing a physical connection between the plasma membrane and the actin cytoskeleton, may lead to marked changes in the general framework of cellular function as well as an aberrant engagement with the extracellular microenvironment, which is directly implicated in metastasis behavior of tumor cells [33]. Thus, it was plausible that the elevated expression of ezrin, connected with the stimulation of tumor invasion and metastasis, may contribute to recurrence and a poorer clinical outcome of osteosarcoma. Kim et al. also revealed that high expression of ezrin in a primary osteosarcoma may directly result in metastasis since ezrin plays a role in multiple metastatic steps such as cell motility, invasion, and adherence [15].

Furthermore, we also observed that patients with positive expression of ezrin had shorter overall survival and poorer metastasis-free survival than those with negative ezrin expression, suggesting that ezrin expression may also be closely linked to poor prognosis of osteosarcoma. One possible explanation could be that ezrin, which is related to the FAK and RhoB, may have a critical role in progression and metastasis in carcinomas and resistance to chemotherapy in osteosarcoma cell lines, and thereby increased expression of ezrin may contribute to worse clinical outcomes of patients with osteosarcoma [33]. Our findings are in accordance with a previous study which found that positive expression of ezrin was distributed in a high percentage of patients with some kinds of osteosarcoma, and all of them had high-grade tumors, indicating that ezrin expression might be an additional prognostic marker in osteosarcoma [14]. However, clinicopathologic factors including gender and age did not have close relationships with the expression of ezrin. To a great extent, our results are in line with previous studies that ezrin expression may have apparent effects on tumor cells metastasis in patients with osteosarcoma and may contribute to poor prognosis in osteosarcoma, suggesting that ezrin expression could serve as a promising biochemical marker for predicting tumor metastasis and survival in osteosarcoma.

RETRACTED

The current meta-analysis also had several limitations that should be acknowledged. First, our results had lacked sufficient statistical power to assess the relationships of ezrin expression with pathological characteristics and prognosis of osteosarcoma due to the small number of studies. Since some of the studies were of a small sample size and even had standard deviations, our meta-analysis may induce fairly wide confidence intervals which restrain our confidence in drawing conclusions. Besides, the small number of studies may constrain the general applicability of our findings, and consequently the cognitive function of our meta-analysis should be considered preliminary. Secondly, meta-analysis is a retrospective study that may lead to subject selection bias and thereby have an impact on the reliability of our results. Thirdly, our meta-analysis failed to obtain original data from the included studies, which may limit further evaluation of the potential role of ezrin expression in the progression and prognosis of osteosarcoma. Although our study has several limitations, this is the first meta-analysis to focus on the correlation of ezrin expression with pathological characteristics and prognosis of osteosarcoma. Furthermore, we performed a highly sensitive literature search strategy for electronic databases. A manual search of the reference lists from the relevant articles was also conducted to find other potential articles. The selection process of eligible articles was based on strict inclusion and exclusion criteria. Importantly, rigorous statistical analysis provided a basis for pooling of information from individual studies.

RETRACTED

To sum up, our results illustrated significant relationships of ezrin expression with pathological characteristics and prognosis of osteosarcoma. Thus, ezrin expression could be a promising marker in predicting clinical outcome of patients with osteosarcoma. However, due to the limitations acknowledged above, larger sample-size works of research with more comprehensive data are required to provide a more accurate and representative statistical analysis.

## Figures and Tables

**Figure 1:** Flow chart shows study selection procedure. Ten cohort studies were included in this meta-analysis.

**Figure 2:** The distribution of the number of topic-related literatures in the electronic database during the last decade.

**Figure 3:** Forest plots for the correlations of ezrin expression with pathological characteristics and prognosis of osteosarcoma.

**Figure 4:** Sensitivity analysis of the summary odds ratio coefficients on the correlations of ezrin expression with pathological characteristics and prognosis of osteosarcoma under the allele and dominant models.

**Figure 5:** Funnel plot of publication biases for the correlations of ezrin expression with pathological characteristics and prognosis of osteosarcoma: a meta-analysis.

**Table 1:** Baseline characteristics and methodological qualities of all included studies.

First author	Year	Country	Ethnicity	Sample	Sample size	Number		Gender (M/F)	Age (years)	Method	NOS score
						Positive	Negative				
Le Guellec [19]	2013	France	Caucasians	36	Small	11	24	19/17	18 (8~57)	LSAB	7
Shen [22]	2008	China	Asians	56	Large	38	18	29/27	22 (7~67)	Envision	8
Salas [23]	2007	France	Caucasians	37	Small	23	14	23/14	15 (7~54)	ABC	7
Kim [15]	2007	Korea	Asians	64	Large	33	31	45/19	19 (4~58)	SP	8
Min [21]	2012	China	Asians	82	Large	49	33	44/38	19 (7~62)	SP	8
Xiong [20]	2011	China	Asians	42	Large	26	16	25/17	42 (10~77)	MaxVision	8
Yang [24]	2010	China	Asians	54	Large	22	32	35/19	23 (12~49)	SP	8
Park [14]	2009	Korea	Asians	31	Small	6	25	15/16	39	ABC	7
Yang [25]	2008	China	Asians	36	Small	20	16	20/16	10~50	SP	7
McHugh [26]	2006	USA	Caucasians	21	Small	11	10	11/10	—	LSAB	6

M: male; F: female; LSAB: labelled streptavidin biotin; ABC: avidin-biotin-peroxidase complex; SP: streptavidin-perosidase.
